# Personalized College English Learning Based on Deep Learning under the Background of Big Data

This article has been retracted.

**DOI:** 10.1155/2022/7361746

**Published:** 2022-06-10

**Authors:** Jingjing Huang

**Affiliations:** Zhejiang University of Science & Technology, Hangzhou, Zhejiang 310023, China

## Abstract

Generally, in-depth learning has been extensively employed in numerous industries to enhance the growth of economic globalization since the dawn of the big data age. At the same time, the demand for foreign language talent has risen dramatically, and more and more businesses are steadily raising their English proficiency standards. International interactions, as well as scientific and technical exchanges, are influenced by English communicating competence. As a result, colleges and universities place a high value on students studying English. However, English learning is also a compulsory course in Colleges and universities, which is different from other courses. Therefore, in setting teaching objectives, arranging teaching activities, and compiling teaching contents, we should highlight students' personalized needs and formulate learning plans in combination with the individual requirements of each student. Aiming at this problem, this paper adopts the deep learning method to study the personalized learning of College English. Deep learning algorithm utilization in the development of college students' English learning reduces teachers' workload and focuses more on students' personalized needs, which is beneficial to teachers' teaching and students' learning. By analyzing the deep learning neural network model, the process of English speech recognition is described, and the characteristic parameters of English speech are extracted. Then compare and explain the characteristics of deep learning and shallow learning, analyze the relationship between them, and clarify the route of deep learning. Finally, the effect of College Students' personalized learning is analyzed by random sampling, and the effect of College English personalized learning based on deep learning is explained from two aspects: listening effect and reading practice.

## 1. Introduction

In the process of studying college English personalized learning, this paper pays attention to the equal status of students and teachers in teaching activities, takes the needs of students' personalized and harmonious development of English as the core, and uses teaching methods to stimulate students' thirst for knowledge and improve students' learning effect. English teaching is infiltration of language and culture. College English learning is to use this language method to strengthen college students' language communication ability and communicative ability [1]. Each student's interests, knowledge structure, student effectiveness, and learning ability are very different. Therefore, during college English teaching, we should improve students' English learning enthusiasm from the perspective of students' personality.

Deep learning is a machine learning and artificial intelligence (AI) technique that mimics how people acquire knowledge. Data science, which also encompasses statistics and predictive modeling, contains deep learning. Deep learning approaches try to learn feature hierarchies composed of lower level features, with features from higher levels of the hierarchy. Without relying only on human-crafted features, a system may learn complicated functions mapping the input to the output directly from data by automatically learning features at several levels of abstraction. DP methodology has been considered as an extremely useful development in the field of AI, and that is the main reason why it has been used in different application areas. DP has been considerably used in the evaluation studies of the student learning objectives and how to improve teaching methodologies.

This paper uses a deep learning algorithm to study college students' Personalized English learning. Through an in-depth understanding of students' English learning situation, this paper analyzes and judges students' learning thinking, reintegrates personalized needs into the previous cognitive structure, and transfers the learned Basic English knowledge in the new situation as a new learning mode to deal with problems and implement decision-making. The cultivation of College Students' deep learning ability is the core goal of cultivating talents in Colleges and universities. Therefore, this paper uses a deep learning algorithm to study college students' Personalized English learning and uses personalized teaching strategies and means to guide and inspire students' English learning.

The main innovations during the research period of this paper are as follows: (1) investigating the deep learning method employed in the personalized learning process of College English during the research period of this work. We can distinguish English speech and extract English pronunciation attributes using this approach. Teachers assess pronunciation using the students' English pronunciation feature information, appraise students' English learning status, and rate each student's English learning level using the data to create a customized English learning plan for them [2]. (2) Comparing and contrasting the features of deep and shallow learning, examining the link between the two, and designing a customized deep learning path for college students. This research examines the tailored learning impact of deep learning [3], starting with the students' listening effect and reading practice.

The remaining manuscript is arranged according to the following agenda items.

In the section “Related work,” summaries of the existing approaches with associated issues are reported. In section 3, English speech recognition based on deep learning in the context of big data is described where various portions such as Artificial neural networks are described in detail. Simulation results are presented where existing and proposed systems are implemented using similar environmental and experimental setups. Finally, concluding points are reported in the last section.

## 2. Related Work

Foreign countries first began to study the theory of deep learning. Erdem and BEKE proposed the concept of shallow learning and deep learning for the first time. They preliminarily analyzed learners' reading process, trained students' deep reading process in an experimental way, and used deep learning to cultivate students' personal hobbies and interests [4]. Prabowo et al. proposed on the research of deep learning that deep learning is an important process of establishing knowledge system, which is conducive to cultivating people's independent thinking ability and helping students better understand life and reading problems [5]. ALT proposes that deep learning is a process of accumulating learning experiences. Using deep learning can strengthen students' learning transfer ability and effectively improve students' learning efficiency [6]. China has a short time to study deep learning. Starting from the field of education, we compare the differences between foreign and domestic deep learning research. Lei *y* established the “SPOC + offline classroom” teaching mode of in-depth learning for College English and offered SPOC experience English for all college students [7]. Chinese He scholars deeply analyze and study the knowledge structure and programmatically transform the knowledge structure into a knowledge structure that can optimize Learners [8]. Zhou comprehensively analyzes deep learning from different perspectives and puts forward that the essence of deep learning is to comprehensively grasp and analyze the learning situation by individuals, and the use of deep learning can transform knowledge in various situations [9]. Jing et al. focus on analyzing the basic content of deep learning and point out that learners can improve their knowledge recognition ability by using deep learning, effectively distinguishing the enthusiasm and negativity of knowledge, and facilitating the better transformation of personal knowledge [10]. Xie and Zhang put forward that teaching management has many characteristics, which mainly embody the following aspects: the advanced nature of teaching philosophy, the scientific nature of courses, the appropriateness of selecting teaching materials, the remarkable teaching methods, the modernity of teaching mode, and so on. [11] Yang and Zhao established the “integration of teaching, learning and management” mechanism from the level of teaching practice and management by using the concept of multilayer governance [12]. The school level should have the scale and perspective of top-level design, and the teacher level should have the management mechanism of incentive, guidance, and supervision. Yang and Wu proposed that the components of the construction of College Students′ English teaching quality assurance system include a teaching condition assurance system, teaching management organization system, teaching quality evaluation system, and teaching process monitoring system. The school, government, and society jointly form an external security system and formulate the maintenance scheme and operation mechanism of the quality assurance system [13]. Wang has proposed that evaluation criteria of students′ application ability must follow the basic principles of fairness, balance, and efficiency and comprehensively use a variety of incentive measures to realize multilevel and multidimensional evaluation and incentive mechanisms [14]. Deep learning allows computational models made up of several processing layers to learn multiple-level data representations. Apart from it, the Keras deep learning package makes it simple to create and analyze neural network models for multilabel classification problems.

## 3. English Speech Recognition Based on Deep Learning in the Context of Big Data

### 3.1. Deep Learning Neural Network Model

An artificial neural network (ANN) uses multiple neurons to connect with each other, simulates the neural information processing mode of the human brain through a neural network, and realizes nonlinear transformation and parallel processing of information [15]. A neural network is used to simplify, abstract, and simulate human brain thinking. A neural network is a set of algorithms that attempts to detect underlying relationships in a piece of data using a technique that is similar to how the human brain works. Neural networks, in this context, refer to natural or artificial systems of neurons. It has nonlinear characteristics, parallel distribution structure, summary, and inductive learning ability. Based on this feature, it can be applied to signal processing, pattern recognition, signal control, time series analysis, and so on. It has become the first choice in commercial and industrial research fields. At present, a neural network is applied in signal processing fields such as compressed speech data, speech analysis, synthetic speech, speech poverty, and speech recognition. As a basic information processing unit, neurons in Ann are called nodes or nodes.  Figure 1 is the schematic diagram of the neuron model [16]:

1. Neurons are made up of connections, and the weights on those connections can indicate their strength of those connections. The value can be either positive or negative, with a positive value indicating inhibition and a positive value indicating activation.
2. An adder that calculates the highlight weighting value corresponding to the input signal.
3. The excitation function can limit the output amplitude of neurons. The excitation function controls the output signal to take value in a certain interval, usually in the [- 1, 1] or [0, 1] interval [17].

In addition, external bias can be added to the neuron model and recorded as *θ*. The bias function is to judge the increase or decrease of the network input of the excitation function according to the positive and negative value. Therefore, the artificial neuron can be represented by the following formulas (1) and (2):

(1) $$\begin{array}{c} a=\sum_{i=1}^{r}\omega_{i}x_{i}, \end{array}$$

(2) $$\begin{array}{c} y=f\left(a+\theta \right). \end{array}$$

The above formula *x*_1_, *x*_2_,…*x*_*r*_ is used to represent *r* inputs on any neuron, and the connection strength of the *i* input is represented by *ω*_*i*_, *θ* represents neuron bias, and *y* represents neuron output. Therefore, the neuron is a nonlinear structure with multiple input structures and a single output.

### 3.2. English Speech Recognition Process

Figure 2 above shows the speech recognition process. First, use PC sound card to digitally convert speech into analog signal to collect speech signals. During the conversion of a digital signal or analog signal based on the Nyquist sampling theorem, if the *f*_s_max_ sampling frequency signal is twice the maximum frequency signal of *F*_max_, the formula is expressed as follows:

(3) $$\begin{array}{c} f_{s\max}\geq 2*F_{\max}. \end{array}$$

After the sampling, the digital signal can represent the effective information in the original voice signal. Generally, the human voice frequency is 40–4000 Hz, so the sampling frequency is set to 8 kHz. This difference in the frequency domain allows communicating activity to be completed in a smooth and sound manner, especially without any interference, and then further preprocess the speech signal. The basic units of speech processing mainly include preemphasis, windowing, framing, and endpoint detection. Secondly, extract the feature parameters on the preprocessed speech signal, process the speech feature parameters by the selection, and complete the model training or matching operation.

### 3.3. Feature Parameter Extraction of English Speech

Basis of auditory excitation. In reality, the response sensitivity of the human ear to speech signals with different frequencies is different, which is similar to the nonlinear system and shows a logarithmic relationship. The MFCC feature parameter extraction process is shown in Figure 3 below.

The following is the basic process of the MFCC speech feature parameter extraction algorithm:

(1) The fast Fourier transform (FFT) is calculated as follows:
  (4) $$\begin{array}{c} X\left[k\right]=\sum_{n=0}^{N-1}x\left[n\right]e^{-j2\pi /Nnk},\;k=0,1,2,\ldots ,N-1. \end{array}$$
Above *X*[*n*],*n* = 0,1,2, ..., *N*−1 is the frame length of a discrete speech sequence *N* obtained after sampling. *X*[*k*] represents a complex sequence on *N* points.
(2) Convert the actual frequency scale to the Mel frequency scale, and its calculation formula is as follows:
  (5) $$\begin{array}{c} \text{Mel}\left(f\right)=2597\mathrm{lg}\left(1+\frac{f}{700}\right). \end{array}$$
In the above formula, Mel (*f*) represents Mel frequency, and *f* represents the real frequency Hz.
(3) By configuring the triangular filter bank, the amplitude spectrum of |*x* [*k*] signal corresponding to the triangular filter is calculated and output by the following formula after filtering:
  (6) $$\begin{array}{c} F\left(l\right)=\sum_{k=f_{0}\left(l\right)}^{f_{h}\left(l\right)}w_{l}\left(k\right)X\left[k\right]\;l=1,2,\ldots ,L. \end{array}$$
(4) Logarithmically operate all filter output results and perform discrete cosine transform (DTC) on them to obtain the following MFCC features:
  (7) $$\begin{array}{c} M\left(i\right)=\sqrt{\frac{2}{N}}\sum_{l=1}^{L}\log\;F\left(l\right)\cos\left[\left(l-\frac{1}{2}\right)\frac{i\pi }{L}\right]\;i=1,2,\ldots ,Q. \end{array}$$
The above formula *Q* represents the order of parameters on MFCC, where the value is 13, and *M*(*i*) represents all parameters of MFCC.

## 4. Personalized College English Learning Based on In-Depth Learning

### 4.1. An Overview of In-Depth Learning

Deep learning, also known as deep learning, was first proposed in the United States. Since then, experts and scholars at home and abroad began to study and explore the theory and practice of deep learning. Deep learning builds a connection between related new learning materials, new concepts, and existing knowledge, transfers or applies the new knowledge learned to different situations, while shallow learning is a learning mode of traditional mechanical memory and recitation. The characteristics between deep learning and shallow learning are listed in Table 1.

Deep learning is used to express that students can deeply develop students′ information during the period of acquiring new knowledge. Students can use new content and new knowledge to carry out in-depth analysis, analyze its connotation, essence, and significance, and form a new teaching mode through continuous analysis, so as to change the previous learning ideas. Students use the way of deepening learning to form self-learning, and in-depth learning is highly relevant. Students must have solid basic knowledge, carry out in-depth mining on this basis, build the connection between various knowledge, and build a complete knowledge framework and structure.

### 4.2. Thinking Structure Level of Deep Learning

Shallow learning is low-level thinking, whereas deep learning is creative and active and belongs to high-level thinking, according to the examination of thinking structure. High-order thinking is one of the primary linkages in deep learning, and it has a direct influence on the achievement of its learning objectives. At the horizontal level, the growth of high-level thinking can actualize the cognition of high-level cognitive capacity and mental activities. A range of high-level cognitive talents, such as synthesis, analysis, creativity, and assessment, are mirrored in the classification of educational objectives. The single classification technique established by educational psychologists is utilized to assess high-order thinking capacity in this research. The grade and feature evaluation approach explains this procedure. It measures the depth of issue knowledge and learning quality by judging cognitive development and cognitive response level in relation to the complexity of learners′ thought structures while dealing with situations [18].  Table 2 shows the meanings of different structural levels in solo classification.

Solo classification is analyzed from the cognitive stage function and solo perspective to explain the development process of learners′ individual cognition. The functional mode abstracts cognitive development, and the solo level has become increasingly complex, indirectly reflecting the improvement of the level of cognitive response. The quantitative change stage of learners′ response level is the development process of prestructure, while the qualitative change process is reflected in the trend from multiple structures to relevance structure and further abstracting relevance structure to expansion structure, indicating that learners′ functional level is higher. Therefore, solo classification can be used in deep learning to evaluate the results of deep learning.

### 4.3. Deep Learning Teaching Mode

Figure 4 shows the deep learning route (DELC). According to the analysis of the map, the components of the route include seven different key points, namely curriculum design and standards, preassessment, learning culture, activation of prior knowledge, learning new knowledge, in-depth processing of knowledge, and evaluation of students′ learning. The above key points are called deep learning strategies [19]. According to the analysis of the chart, there are two ways of evaluating students′ learning to acquiring new knowledge. First, teachers evaluate and analyze students′ learning, complete standard design and curriculum planning, preevaluate students′ curriculum research and learning status, design preclass guidance, and then activate students′ previous knowledge, and then impart new knowledge [20]. Another way is to analyze from the perspective of evaluating students′ learning so as to help students learn new knowledge by means of deep processing. This paper constructs the teaching mode of College Students′ in-depth learning under the Enlightenment of the road map, as shown in Figure 4 below.

## 5. Analysis of Personalized Learning Results of College English Based on Deep Learning

In the context of big data, this paper studies the personalized learning of College English based on deep learning, formulates a deep learning route for college students, and applies it in Colleges and universities. After a one-year citation, 1000 college students were randomly selected by systematic random sampling, and then 50 students′ listening and reading scores were selected from the 1000 students as the research objects to analyze college students′ Personalized English learning achievements.

### 5.1. Analysis of Listening Effect of Personalized Learning of College English

Firstly, this paper analyzes the effectiveness of the randomly selected student sample data and uses the method of calculating the average difference to process the sample data. The basic process is to select the first two scores as the initial scores and the last two consecutive scores as the final scores. The improvement degree of each score can be obtained by subtracting the final score from the initial score.  Figure 5 below shows the growth of College Students′ listening scores.

The data in Figure 5 shows that among the 50 randomly selected students, 63% have improved their scores by 10–25 points, 15% have improved their listening scores by more than 30 points, and only one has increased their listening scores by 55 points, indicating that most students have achieved significant improvement in their listening scores after using the personalized College English learning method based on deep learning. This part only makes a statistical analysis on the growth of students′ performance. In addition, 10 students′ performance is selected as a sample in listening practice so as to better grasp the actual practice status of learners.  Figure 6 shows the listening practice of college students.

We can observe from the listening practice statistics in Figure 6 that kids have a lot of listening practice. The average number of hearing practice sessions per month is 18 to 30, and listening performance varies widely; yet, most students feel that listening is the most difficult portion of the English test. Therefore, they practice listening more.

### 5.2. Analysis of Reading Results of Personalized Learning of College English

Figure 7 shows the score increase of the reading practice effect.

According to the histogram in Figure 7 above, 65% of students′ reading analysis scores increased by 10 to 25 points, and 16% of students did not increase or even decrease significantly after using the personalized learning mode of college students. Students′ reading scores improve faster, but there is still a large number of students' reading scores that have not increased significantly. By analyzing the above reading performance increase, most students' performance increase is relatively concentrated. After the increase exceeds 45, the number decreases. Only one person's reading score increases by 60 points. After calculation, the reading score increase is about 45 points, and the students' reading practice is shown in Figure 8 below.

According to the reading exercises shown in Figure 8 above, the average number of reading exercises per month is 10–30. Students' reading ability has been significantly improved after personalized learning. After each practice, the reading performance of college students has improved to a certain extent, which shows that after personalized learning, students have the stronger initiative in English learning, can actively carry out English reading training, and have a strong interest in English learning.

## 6. Conclusion

The amount of data created every day has increased dramatically since the dawn of the big data era. People are having difficulty locating useful and high-value data in these databases. The deep learning algorithm is used to solve this problem since it can mine and analyze all types of data and extract important information, which is beneficial to the growth of many enterprises. Deep learning is now widely applied in many aspects of society. In this paper, we have extensively utilized a well-known approach, i.e., deep learning analysis, when studying college students' English personality learning. Deep learning belongs to the current efficient learning mode. Using deep learning can improve students' mastery of knowledge structure, adjust students' thinking mode and way of thinking, and understand deeper knowledge. In the process of College Students' Personalized English learning, we should use the deep learning method to excavate students' characteristics, clarify each student's English level and personalized needs, formulate application learning plans that meet their requirements, and realize personalized English teaching. This method is conducive to the development of teachers' teaching, and students can obtain more English knowledge. This paper analyzes the improvement of students' listening and reading performance after using personalized teaching. The results show that 63% of students' scores in listening are improved by 10 to 20 points, 15% of students' scores are improved by about 30 points, 65% of students' scores are improved by 10 to 25 points, and the number of students whose scores have not increased or decreased slightly accounts for about 16%. The overall analysis shows that about 80% of the students have significantly improved their scores after taking personalized learning, while the improvement of listening scores is slower than that of reading.

## Figures and Tables

**Figure 1:** Schematic diagram of the neuron model.

**Figure 2:** Speech recognition process.

**Figure 3:** MFCC feature parameter extraction process diagram.

**Figure 4:** Deep learning route.

**Figure 5:** Growth of college students′ listening performance.

**Figure 6:** Listening practice.

**Figure 7:** Reading exercise score increase histogram.

**Figure 8:** Reading practice.

**Table 1:** The characteristics of deep learning and shallow learning.

	Deep learning	Shallow learning
Memory	Deep understanding and active learning	Mechanical and repetitive memory knowledge
Reflect on state	Reflect and learn from relevant information	Lack of flexibility in learning methods
The focus	Start from the whole macro analysis, long-term consideration	Strong vision limitations and attention to details
Learning motivation	Learning is driven by interest	Fear of failure as the main driving force of learning
The knowledge system	Integrate existing knowledge with new knowledge	Seamless connection between past knowledge and new knowledge
Ability to migrate	Deal with practical problems in combination with personal experience	Effectively separate personal ability and knowledge
Input level	Collect and learn to expand knowledge content	Do not accumulate content that is not related to knowledge
Thinking level	Higher-order thinking	Low order thinking

**Table 2:** SOLO taxonomy hierarchy.

Solo hierarchy	Concept description
Anterior structure	Learners complete learning tasks together. However, due to the existence of a large number of other knowledge in the learning situation, they are misled in the learning process
Single structure	Students only analyze the knowledge and information related to problem handling
Multivariate structure	Students use multiple separate knowledge information to deal with problems, lack certain integration abilities, and do not build links between different knowledge
Association structure	Students can integrate various knowledge information, construct the connection between different knowledge information, and form a complete knowledge structure for dealing with complex problems
Abstract structure	Based on relevance thinking and analysis, learners summarize and analyze the characteristics of abstract paintings, form hypotheses, use them in a new environment, and expand their own value

## Data Availability

The datasets used and/or analyzed during the current study are available from the corresponding author upon reasonable request.
